# Vehicle Driving Risk Prediction Model by Reverse Artificial Intelligence Neural Network

**DOI:** 10.1155/2022/3100509

**Published:** 2022-10-07

**Authors:** Huizhe Ding, Raja Ariffin Raja Ghazilla, Ramesh Singh Kuldip Singh, Lina Wei

**Affiliations:** ^1^Centre of Product Design and Manufacturing, Department of Mechanical Engineering, Faculty of Engineering, University of Malaya, Kuala Lumpur 50603, Malaysia; ^2^School of Mining and Geomatics, Hebei University of Engineering (Hebei), No. 19 Taiji Road, Handan Economic and Technological Development District, Handan 056038, China

## Abstract

The popularity of private cars has brought great convenience to citizens' travel. However, the number of private cars in society is increasing yearly, and the traffic pressure on the road is also increasing. The number of traffic accidents is increasing yearly, and the vast majority are caused by small private cars. Therefore, it is necessary to improve the traffic safety awareness of drivers and help car manufacturers to design traffic risk prediction systems. The Backpropagation neural network (BPNN) algorithm is used as the technical basis, combined with the MATLAB operation program, to simulate the driving process of the car. Dynamic predictive models are built to predict and analyze vehicle safety risks. Multiple experiments found that: (1) in various simulations, the simulation driving process of MATLAB is more in line with the actual car driving process; (2) the error between BPNN and the actual driving prediction is within 0.4, which can meet the actual needs. Predictive models are optimized to deploy and predict in various traffic situations. The model can effectively prompt risk accidents, reduce the probability of traffic accidents, provide a certain degree of protection for the lives of drivers and passengers, and significantly improve the safety of traffic roads.

## 1. Introduction

With the continuous development of social science and technology, automobiles play a major role in traffic travel. Traffic accidents have caused widespread concern, seriously threatening the safety of human life and property [1]. Statistics show that about 1.2 million people are killed in traffic accidents every year around the world. Driver factors cause about 80% of tragedies. Bad driving behavior will cause great discomfort for passengers and even cause psychological pressure on drivers [2]. The driver needs to process the information in time while receiving the traffic information while driving, and the driving risk is everywhere. Safe driving requires drivers to maintain a vigilant attitude in driving [3].

There are numerous studies on the relationship between drivers and traffic accidents, but few studies on the risk warning of the vehicle itself. According to the basic physiological and psychological characteristics of drivers, combined with the specific functions of the car, the prediction of traffic risk is an emerging topic [4]. An artificial neural network (ANN) is a multilevel early-warning model, which uses data analysis technology to predict driver behavior and system, showing strong flexibility and adaptability [5]. The BPNN can perform correlation analysis on multiple complex relationships, make macro predictions of accidents, reduce the risk of accidents, and provide security [6].

First, a simulation driver system based on the MATLAB computer program is proposed. Dynamic simulation models are built to perform dynamic analysis of vehicle driving. Second, the BPNN is used to build different structures and analyze driving safety risk and accident prediction. The driver's association with accident occurrence is explored. Finally, combined with the error backpropagation algorithm, different experimental data are detected, recorded, and compared. Driving safety risks and effective countermeasures are analyzed. This work intends to study the relevant factors of car accidents during driving, reduce the risk index of driving safety in people's travel and traffic, give early warning of possible accident risks, and conduct research. It is committed to reducing and preventing driving errors from the root cause and effectively improving the status quo of road traffic safety.

## 2. Materials and Methods

### 2.1. Realization and Simulation of Driving Simulation in MATLAB

Today, in the automotive industry, it is planned to use computer simulation to integrate more real system data, various machine plate components, and electronic control units into the vehicle model to develop and operate various types of automotive products. Research in this area has become one of the hot spots [7]. The operation of the internal electronic control system and mechanical dynamics of the automobile requires the use of related technologies to simulate the transient motion process of the automobile. The actual motion state process of the car is shown in Figure 1.

#### 2.1.1. Simulation Environment

MATLAB software has been widely used in the design and simulation of control systems. At this stage, the field of simulation technology is a relatively mature scientific computing language, which is good at efficiently processing large amounts of data and visualizing data [8]. MATLAB is used to simulate the driving process of the car and analyze how the car engine and clutch, and other components break and operate in an emergency. The control system is simulated, and the risk factors affecting the driving control system of the vehicle are obtained more intuitively, which provides a strong scientific basis for the risk estimation and performance improvement of the vehicle in the future. MATLAB software is used to simulate the car driving system. The frame line of the car simulation driving system is shown in Figure 2.

Figure 2 is the frame line of the car simulation driving system. First, we open the window of the car simulation driving system and input various parameter values required for simulated driving, including the number of gears of the transmission, the number of front-wheel rotation angles, and the degree of throttle opening. [9]. The system will match the corresponding actual road conditions on the ground according to the different scenarios selected and import it into the dynamic simulation system of the car as the parameters to be matched later. After matching, the system performs dynamic simulation and presents the results with virtual technology. When different scenarios are selected to be simulated again, only the parameters of the car driving system need to be changed [10].

#### 2.1.2. Mathematical Model of the Algorithm

In the vehicle driving speed control system, the position transmission belongs to the speed manipulation tool and is the main input part of the system. Its functions mainly include reasonable control of the speed and transition of car driving, as shown in the following:

(1) $$\begin{array}{c} v=ax+b,x\in \left[0,1\right], \end{array}$$

*x* represents the position of the speed control mechanism; *v* represents the driving speed corresponding to it; and *a* and *b* represent constants.

In the vehicle control system, proportion-integral-derivative (PID) belongs to the core part, which mainly compares the current speed of the car with the speed at which it is specified. The difference between the two speeds is the current vehicle traction [11]. The calculation of the driving controller is shown in equations (2)-(4)as follows:

(2) $$\begin{array}{c} \text{Calculus equation part}:x\left(n\right)=x\left(n-1\right)+u\left(n\right), \end{array}$$

(3) $$\begin{array}{c} \text{Differential equation part}:d\left(n\right)=u\left(n\right)-u\left(n-1\right). \end{array}$$

(4) $$\begin{array}{c} \text{The output section of the system}:y\left(n\right)Pu\left(n\right)+Ix\left(n\right)+D\;d\left(n\right), \end{array}$$

*u*(*n*) represents the system input value, that is, the difference between the current speed of the car and the specified speed; *y(n)* represents the system output value, representing the traction force of the car; and *x(n)* represents the state of the system.

In the vehicle driving control system, the vehicle power mechanism belongs to the actuator. Its function mainly uses the traction force to change the vehicle's speed so that the speed is the same as the specified value. The mathematical expression between traction and speed is *F*=*mv*+*bv*. *F* represents the traction force generated by the car; *m* represents the mass of the car; *v* represents the speed of the car; and *b* represents the drag factor of the car [12].

#### 2.1.3. Parameter Setting

After opening the MATLAB interface, we enter the relevant parameter values in the GUI interface. Simulink's default simulation time is 10 seconds. In the initial stage of the engine, there is a certain initial speed, which is set to 2000 n/min [13]. The car is running at a constant speed at this stage. We accelerate and apply the brake while the car is driving at a constant speed. The specific parameter value settings are shown in Table 1.

According to the operation of the actual vehicle starting process, MATLAB simulation software is used to establish the simulation model of vehicle starting. The model includes four plates: engine, transmission, body, and road resistance plates [14]. According to the modeling idea of the simulation model, the complex molecules in the system are subdivided into smaller plates. The vehicle driving simulation model is shown in Figure 3.

In Figure 3, after the simulation model is built, the simulation parameters are set according to the system requirements. The position transmission part of the speed control mechanism adopts the Slider Gain module. It can limit the range of the input signal *x* of the position transmission. Among them, the parameter minimum value is set to 0, the maximum value is set to 1, and the initial value is set to 0.55. In the Gain module, the gain value is set to 50. In the Constant 1 module, the constant value is set to 45. In the vehicle powertrain subsystem model, the Gain module is adopted, its value is 1/m, and the specific value is 1/1000. The value of the Gain 1 module is b/m, and the specific value is 20/1000. The automotive powertrain adopts the Integrator integral module. The initial state is set to 0, which is the initial speed value of the car. In the driving controller subsystem model, the Delay block is used to implement the PID controller, the initial state is set to 0, and the sampling time is set to 0.02 s. The simulation time range of the system is set from 0 to 500 s. The variable-step continuous solver is selected. The rest of the other modules and simulation parameters use MATLAB default values [15].

## 3. ANN

Based on the basic characteristics of artificial intelligence to simulate the brain of living things, a new network model ANN is proposed. It can simply simulate and simplify different biological networks and provide help for the research of various functions of the real biological brain nervous system. The basic components of ANN include neurons and synapses. Among them, the function of a neuron is called a processing unit, which can use digital language to express the information processing method of the biological neuron, formally describe the biological neuron, and simulate the function and function of the expression structure [16].

### 3.1. Structure of an Artificial Neuron

An artificial neuron is an abstract concept of a biological neuron. The transmission of signals between neurons is also a transmission of values. Multiple signals are received and then converted into a new round of signals to be transmitted, which belongs to a nonlinear structure. The specific structure is shown in Figure 4.

Figure 4 shows the structural model of an artificial neuron, which is seen as a simple processor that performs a weighted summation of incoming signals. The specific description is shown in the following:

(5) $$\begin{array}{c} Y=W_{0}+W_{1}X_{1}+W_{2}X_{2}+\ldots +W_{m}X_{m}. \end{array}$$

In equation (5), (*X*1), (*X*2),…, *X*_*m*_ represent the input value; *W*_1_, *W*_2_,…, *W*_*m*_ represent the weights corresponding to the input value, that is, the synapse of the simulated neuron; *Y* represents the output of the neuron; and *W*_0_ represents the system bias.

The network composed of artificial neurons is ANN. Since the emergence of this theory, it has been continuously improved, and now a relatively complete theory has been formed, which is widely used in different fields [17]. The application research of neural networks in traffic safety risk warning is based on the practical application background of the deep learning theory, combined with the actual driving situation, analyzes the possibility of vehicle risk in some cases, and carries out early warning according to the operation mechanism of the neural network, so as to reduce the possibility and harm of traffic accidents [18].

### 3.2. Establishment of the Risk Assessment Model

There have been many attempts at applying ANN in risk assessment. Many practices have confirmed that it is a better risk assessment method and can be used as a supplement to traditional risk assessment. The system can analyze the risk assessment with the law of actual risk occurrence and provide a basis for the early-warning system. An ANN risk assessment model is proposed, as shown in Figure 5.

Based on ANN, a risk model for driving safety is established. The practical application is divided into six steps. (1) The number of layers in the middle hidden layer of the neural network is determined, including the number of input, output, and hidden layer nodes. (2) Characteristic parameters and state parameters are determined. In the process of risk analysis, the internal structure and external parameters in the risk assessment system are determined, and it is ensured that the results and state characteristics of the input parameters can be correctly reflected. (3) The neural network system needs to provide a variety of learning samples for feedback learning during execution and analyze the network system for parameter values in different states. This process is that the neural network determines the connection weights and errors of the network system according to the selected samples. (4) The nonlinear sigmoid function is chosen as the action function. (5) Network learning is used to confirm the structure of the neural network to establish a knowledge base for risk analysis of the nervous system so that the evaluation system has certain inference and prediction functions. (6) The actual driving situation is analyzed. The actual eigenvalues of the system that have been calculated are input into the neural network with a prediction function. After the data are processed by the internal risk assessment system, the evaluation results are obtained. Additionally, this result is fed into the neural network as a new computational sample, which enriches the risk assessment system database [19].

## 4. BPNN Model

### 4.1. The Principle of BPNN

The BPNN is a multilayer feedforward network trained according to the error backpropagation algorithm, and it is one of the most widely used neural network models. It can learn and store many input-output relative relationships without revealing the mathematical equations describing this mapping in advance. The learning method of BPNN uses the steepest descent method and backpropagation to repeatedly modify the weights and thresholds of the system to minimize the sum of squared errors [20]. The BPNN structure includes three parts: input, hidden, and output layers. The specific structure is shown in Figure 6.

In Figure 6, the operation process of BPNN consists of two parts: forward propagation of data and backpropagation of error. During forward propagation, data are passed in from the input layer. After passing through the hidden layer, it is passed out from the output layer. If the actual output situation of the output layer is different from the ideal output, the result turns to the backpropagation stage of the error [21]. The backpropagation of the error means that the output error enters the hidden layer in a certain way and is transmitted back to the input layer, and the error data are apportioned to all units of each layer to obtain the error data of each layer unit. These error data are used as the basis for correcting the weights of each unit [22]. The BPNN consists of input, output, and hidden layers. N_1_ is the input layer, *N*_m_ is the output layer, and the rest are hidden layers.

### 4.2. Algorithm Derivation of Backpropagation Three-Layer Neural Network

During the forward propagation, the activation function of neuron *j* produces the induced local domain *V*_*j*_*(n)* at the input, as shown in the following:

(6) $$\begin{array}{c} v_{j}\left(n\right)=\overset{m}{\underset{i=0}{\sum }}w_{ji}\left(n\right)y_{i}\left(n\right). \end{array}$$

∅_*j*_ is the activation function. The representation of the function signal *y*_*j*_(*n*) at the output of neuron *j* is shown in the following:

(7) $$\begin{array}{c} y_{j}\left(n\right)=\varphi_{j}\left(v_{j}\left(n\right)\right). \end{array}$$

In the process of error backpropagation, *y*_*j*_(*n*) represents the actual output of neuron *j*; *d*_*j*_(*n*) represents the expected output of neuron *j*, which is the *j*-th element of the expected response vector *d*(*n*). The error signal *e*_*j*_(*n*) is shown in the following:

(8) $$\begin{array}{c} e_{j}\left(n\right)=d_{j}\left(n\right)-y_{j}\left(n\right). \end{array}$$

Minimizing the root mean square error makes the function continuously differentiable. Here, the instantaneous error energy of neuron *j* is given, as shown in the following:

(9) $$\begin{array}{c} E_{j}\left(n\right)=\frac{1}{2}e_{j}^{2}\left(n\right). \end{array}$$

The error energies of all output layer neurons are summed up, i.e., the sum of the instantaneous error energies of the entire network is obtained, as shown in the following:

(10) $$\begin{array}{c} E_{n}=\underset{j\in C}{\sum }E_{j}\left(n\right)=\frac{1}{2}\underset{j\in C}{\sum }e_{j}^{2}\left(n\right). \end{array}$$

In equation (10), set C refers to all neurons in the output layer.

The backpropagation algorithm minimizes *E*_*n*_ by modifying the weights multiple times. The iterative gradient descent method is used to apply a correction value ∆*w*_*ji*_(*n*) to the synaptic weights *w*_*ij*_(*n*). It is proportional to the partial derivative *δE*(*n*)/*δw*_*ji*_(*n*). According to the differential chain method, this gradient is given by the following:

(11) $$\begin{array}{c} \frac{\partial E\left(n\right)}{\partial w_{ji}\left(n\right)}=\frac{\partial E\left(n\right)}{\partial e_{j}\left(n\right)}\frac{\partial e_{j}\left(n\right)}{\partial y_{j}\left(n\right)}\frac{\partial y_{j}\left(n\right)}{\partial v_{j}\left(n\right)}\frac{\partial v_{j}\left(n\right)}{\partial w_{ji}\left(n\right)}. \end{array}$$

The partial derivative *δE*(*n*)/*δw*_*ji*_(*n*) represents a sensitive factor, which determines the search direction of the synaptic weight *w*_*ji*_(*n*) in the weight space.

(12) $$\begin{array}{c} \frac{\partial E\left(n\right)}{\partial e_{j}\left(n\right)}=e_{j}\left(n\right), \end{array}$$

(13) $$\begin{array}{c} \frac{\partial e_{j}\left(n\right)}{\partial y_{j}\left(n\right)}=-1, \end{array}$$

(14) $$\begin{array}{c} \frac{\partial y_{j}\left(n\right)}{\partial v_{j}\left(n\right)}=\varphi_{j}^{\prime }\left(v_{j}\left(n\right)\right), \end{array}$$

(15) $$\begin{array}{c} \frac{\partial v_{j}\left(n\right)}{\partial w_{ji}\left(n\right)}=y_{i}\left(n\right). \end{array}$$

Equations (7)-(10) are substituted into equation (6), as shown in the following equations (16) and (17):

(16) $$\begin{array}{c} \frac{\partial E\left(n\right)}{\partial w_{ji}\left(n\right)}=-e_{j}\left(n\right)\varphi_{j}^{\prime }\left(v_{j}\left(n\right)\right)y_{i}\left(n\right), \end{array}$$

(17) $$\begin{array}{c} ∆w_{ji}\left(n\right)=-\eta \frac{\partial E\left(n\right)}{\partial w_{ji}\left(n\right)}. \end{array}$$

∆*w*_*ji*_(*n*) is the correction function of *w*_*ji*_(*n*); *η* represents the learning rate of error backpropagation; the negative sign represents gradient descent. Equation (11) is substituted into equation (12), as shown in the following:

(18) $$\begin{array}{c} ∆w_{ji}\left(n\right)=\eta \delta_{j}\left(n\right)y_{i}\left(n\right). \end{array}$$

In equation (18), *δ*_*j*_(*n*) is the local gradient defined according to the delta law. It indicates the required changes in synaptic weights, as shown in the following:

(19) $$\begin{array}{c} \delta_{j}\left(n\right)=-\frac{\partial E\left(n\right)}{\partial e_{j}\left(n\right)}\frac{\partial e_{j}\left(n\right)}{\partial y_{j}\left(n\right)}\frac{\partial y_{j}\left(n\right)}{\partial v_{j}\left(n\right)}=e_{j}\left(n\right)\varphi_{j}^{\prime }\left(v_{j}\left(n\right)\right). \end{array}$$

### 4.3. Algorithm Flow of BPNN

The backpropagation three-layer neural network has been recognized by the public as the most suitable model for simulating input, output, and early warning [23]. The specific operation process is shown in Figure 7.

In Figure 7, the algorithm operation process includes forward and backward propagations. During forward propagation, information data enter from the input layer and are processed by the hidden unit to the output layer. The state of a neuron in each layer only affects the state of neurons in the layer below it [24]. If the output layer does not get the desired result after a series of operations, the data are transmitted back to the backpropagation, and the error signal is returned along the original neuron connection path. When returning, the weights of the neuron connections will be modified one by one [25]. This process is iteratively processed. Finally, the signal error value is within the allowable range. Eventually, the output value is close to the desired output.

## 5. Tips for Traffic Risk Information

There may be latent risk information in the static and dynamic information of traffic. Information that may lead to risk events is risk information. In China's urban road environment, with mixed and nonmotor vehicles, the risk information is mainly motor vehicles, nonmotor vehicles, and pedestrians. There may be latent risk information in the static and dynamic information of traffic. If the response to avoid the risk information is not made in time, it will lead to risk events. Risk events can lead to traffic conflicts, and traffic conflicts can lead to traffic accidents, as shown in Figure 8.

In Figure 8, when the risk information appears, the driver's physiological and psychological factors significantly impact the reaction speed, including the influence of factors such as age, gender, personality, and education level. In addition, the driver's sensitivity to risk information, judgment ability, and feedback speed during driving are also related to the type of risk information. During the driving process, people or things that affect the normal driving trajectory and driving speed of the vehicle can become risk information. In addition to common people and vehicles, there may also be sediment, falling rocks, animals, and poultry on various mountain roads or country trails. The risk information mainly includes pedestrians, nonmotor vehicles, and motor vehicles.

The risk warning model must be consistent with the level of human security risk perception before it can be accepted in practical applications. During the driving process, the driver subjectively feels the changes in the information of the road segment and has a stress response to the information of hidden risks, which is a comprehensive performance. For example, when a driver suddenly encounters a pedestrian crossing the road in front of him, illegally climbing over the guardrail, or the car in front of him suddenly braking, suddenly changing lanes, and so on in normal driving, the driver needs to pay attention and discover the risk information in time in advance. The driver's skills can respond to the predicted risk information and take actions such as braking or steering in advance to avoid dangerous situations.

Therefore, analyzing the driver's perception ability of risk information is the premise of designing a risk early-warning system. Driving a vehicle is an acquired skill that grows with driving experience. An ideal risk warning system should be able to reach or be better than a skilled driver's ability to perceive risks. Otherwise, if the system cannot perform better than the driver, it will lose the meaning of assisted driving. Studies have shown a big difference in driving stability between experienced and novice drivers. This experiment will quantify the driver's perception of risk to provide an effective risk warning threshold for the risk warning system. The architecture of the early-warning system based on radar sensing technology at this stage is shown in Figure 9.

Figure 9 shows the composition and architecture of the vehicle-mounted early-warning system. Laser sensors and other sensing devices collect information such as speed, acceleration, and position and upload them to the central processor for data integration and processing. The system calculates the alarm distance according to the designed early-warning model. Then, the central processing unit sends instructions to the signal output device to promptly and effectively remind the driver through sound and light on the display screen, alarm, and warning lights.

## 6. Results and Discussion

### 6.1. Analysis of the Output of the Model

When a simulator drives a car, the speed display is one indicator of the accuracy of the simulation. Different places have different requirements in the driving speed test of the car. The car's speed should be 30–60 km/h when driving in an urban area. The traffic flow in the urban area is large, and there are many people, so the speed should not be too fast, generally at a constant speed of 40 km. The road surface of the expressway is relatively smooth and belongs to the fast lane, and the speed is generally 80–120 km/h. The road arrangement in this experiment is relatively remote for safety reasons; the traffic flow is small; and the road is smooth, so it is a relatively normal speed to maintain the vehicle speed at 60–80 km/h. Figures 10–13 show the driver's speed change based on the MATLAB simulation driving environment:

Figure 10 shows the score fluctuation of the longitudinal and horizontal speed of the simulated car under the acceleration state. The longitudinal speed has been in a state of steady growth, and the speed value is between 60 km/h and 70 km/h, which is in line with the car's speed in the actual driving process. The lateral speed fluctuates greatly, the speed is controlled below 50 km/h, and the numerical instability factor is too strong. The simulation is in good agreement with the actual situation.

Figure 11 compares the longitudinal and lateral accelerations of the simulated car under the acceleration state. The longitudinal acceleration fluctuates less than the lateral acceleration, and the acceleration value fluctuates up and down at 5 m/s^2^ and is always higher than the lateral acceleration value. The lateral acceleration value is negative, and the value is between −5 and 0 m/s^2^. Additionally, its instability is also high. The state displayed by the data is more in line with the actual driving situation of the car.

Figure 12 is a comparison of the driving speed of the simulated car under braking. The longitudinal speed has been in a state of steady deceleration, and the value is controlled between 20 km/h and 40 km/h. The lateral speed fluctuates up and down. The situation is like the driving speed in the acceleration state. It fluctuates erratically below 20 km/h, and the lateral speed value is always lower than the longitudinal speed value. The state displayed by the data is more in line with the actual driving situation of the car.

Figure 13 compares the acceleration of a simulated car under braking. The value of longitudinal acceleration varies less than that of lateral acceleration, and the deceleration value is controlled from −5 to 0 m/s^2^. When braking, the deceleration value is always lower than the lateral acceleration value, and the situation is relatively stable. The lateral deceleration value fluctuates around 0 m/s^2^, and the instability is strong, which is more in line with the actual driving situation.

Among the driver's speed change values obtained by MATLAB's simulation of the driving environment, the simulation results are like the actual driving conditions of the car and have a high degree of coincidence. In the parameter value debugging process, the stability of the model is relatively good, which meets the simulation requirements. Additionally, in terms of data processing, there are relatively few comparisons of models. The car's driving conditions under acceleration and braking are compared and analyzed. The application of MATLAB in the computer simulation driver needs more practical analysis to ensure that it can be widely used in driving safety risk analysis.

## 7. Risk Analysis of Driving Safety Based on ANN

This paper uses an ANN model to train driving behavior, resulting in multiple individual networks. Then, the neural network dynamic integration algorithm is used for integration to establish a driving behavior model that is closer to the actual situation. The output result is the maximum weighted average of each corresponding neuron in the individual network alliance, which is the output of driving behavior. The error values of the output and the actual situation are compared. The accuracy and optimization scheme of the neural network algorithm is derived. The data results are shown in Figure 14.

Figure 14 is the output comparison between the BPNN simulation result and the actual value. The actual operating values of the driver are simulated. After the input signal value in the network undergoes algorithm operation and program transformation, the neural network model obtains a series of data. Compared with the actual value, the error between the two is analyzed.

The error range between the BPNN simulation results and the actual value is about 0.4, and the error value is relatively low. The data show that ANN can predict and track data to a certain extent in the process of driving safety risk assessment and effectively reduce risks in actual driving safety.

The ANN dynamic ensemble learning method is used to learn driving preferences from historical driving behavior records and save them to the data system to solve the nonlinear relationship between the driving environment and driver behavior. The driving behavior is pretested in terms of the opening degree and time of the driver stepping on the brake pedal and the accelerator pedal, and the steering wheel angle and time. A possible risk indication is drawn from the historical database, and an early warning is issued. The results are consistent with the overall trend of the sample data and reflect the personality of driving behavior. Therefore, when the ANN algorithm is actually applied to driving safety risk analysis, the driver's historical driving behavior should be recorded in the early stage and stored in the database. In this way, after the corresponding situation occurs, more accurate warning prompts can be issued to ensure drivers' safe driving and road traffic.

The research is limited to the theoretical and simulation level and lacks actual data support. There are few mature theories in domestic research in this area, so the established model is still far from the actual situation. The experimental simulation data in the driving behavior research come from the driving simulator, not the data collected on the spot, and the situation of the early-warning system in the actual application process lacks verification. Therefore, the next step is to get out of the simulator, try to collect real driving behavior and driving environment data, and establish a driving behavior and a road condition database for driving behavior learning, so that this research has high practical value.

## 8. Conclusions

In road driving, the driver operating system is multichannel and nonlinear. The MATLAB driving simulator is used to analyze the car's dynamic characteristics during driving and the possible factors of risk occurrence. Combined with the simulated driving environment and the speed change value of the driver, the simulation results are like the actual driving conditions of the car, with a high degree of coincidence. In the parameter value debugging process, the stability of the model is relatively good, which meets the simulation requirements.

The application of ANN in driving safety risk warning is combined with an example of risk prediction. Deep learning, combined with the actual driving situation, analyzes the possibility that the car may have a risk in some cases and issues an early warning based on the ANN operating mechanism to reduce the possibility and injury of traffic accidents. The BPNN is used to model the behavioral characteristics of drivers. The neural network system is practiced and trained many times. The test results are compared with the driver's actual risk value. The error range between the BPNN simulation results and the actual value is about 0.4, and the error value is relatively low. The BPNN model can track the changes of different instructions very well. For imminent hazards, the model warns the driver and exhibits certain predictive and data-tracking capabilities.

Additionally, the data processor also showed certain shortcomings. There are relatively few comparisons of the models. This work only compares and analyzes the driving situation of the car under acceleration and braking state. In the later stage, MATLAB needs to do more practical analysis on the application of computer simulation drivers to ensure that it can be widely used in driving safety risk analysis.

## Figures and Tables

**Figure 1:** The flow of the motion state of the car.

**Figure 2:** The simulated driving frame of the car.

**Figure 3:** Simulation model of car driving.

**Figure 4:** The nonlinear structure of an artificial neuron.

**Figure 5:** ANN's risk assessment model.

**Figure 6:** The structure of BPNN.

**Figure 7:** The flow of the BP algorithm.

**Figure 8:** Relationship of traffic events.

**Figure 9:** Radar-based vehicle conflict warning system.

**Figure 10:** Driving speed under acceleration.

**Figure 11:** Driving acceleration under acceleration.

**Figure 12:** Driving speed under braking.

**Figure 13:** Driving acceleration under braking.

**Figure 14:** Comparison of output results.

**Table 1:** Basic parameter values.

Road slope	Adhesion coefficient	Initial speed n	Throttle opening	Steering wheel angle	Brake percentage	Gear
0.05	0.8	66.7	0.7	0.0	0.0	2

## Data Availability

All data used to support the findings of the study can be obtained from the corresponding author upon request.
